RETRACTED

# A Multimodal Model for College English Teaching Using Text and Image Feature Extraction

**DOI:** 10.1155/2022/3601545

**Published:** 2022-08-16

**Authors:** Dan Zhao, Yafang Liu

**Affiliations:** Institute of Humanities and Education, Xijing University, Xi'an 710123, China

## Abstract

The rapid development of the internet and multimedia technology in recent years has continued to push foreign language education in the direction of modern education. Multimodal education is becoming more and more important in the field of English education as an advanced educational concept in the field of language education. As a result, many English teachers have begun to emphasize the use of multimodal teaching theory in their classrooms. This paper investigates a multimodal model that incorporates text and image features, based on multimodal discourse theory, systemic functional linguistics theory, and foreign language teaching theory. This paper develops a multimodal model that can search for images and texts from various perspectives. We use an image feature bias term in the log-bilinear natural language model to influence the probability of predicting the next word based on the context, resulting in a multimodal model. The experimental results show that the proposed model, as an image-text relationship evaluation index system, has a slower search speed than other models but better search accuracy.

## 1. Introduction

Modality means the interaction with the external environment through visual, auditory, and other sensory systems in the process of human cognition of external things. In the process of this activity, human beings apply language, sound, action, and other means and language symbols to form the analysis of multimodal discourse. The so-called multimodal discourse analysis is to combine social semiotics with a variety of theoretical knowledge such as system function and method, and to regard language as a social symbol, while pictures, body movements, and music can be regarded as a nonverbal symbol expressing image meaning. The combination of the two forms a multimodal form. Text, image, audio, video, and other types of data are expanding at an exponential rate thanks to the quick development of internet technology. Multimodal data [1] present the same event or theme from various perspectives, enhancing people's comprehension of it. A hot topic for research in the field is how to efficiently use multimodal data to carry out the designated tasks in the corresponding scene [2]. With the rapid advancement of deep learning technology in recent years [3–5], people are increasingly able to solve more challenging machine learning problems and have made significant strides in the analysis and processing of multimodal data. Users find it challenging to efficiently and accurately retrieve the information they are interested in due to the growth of multimodal data. As of right now, the first practice test is based on single modalities, such as text, image, or multimodal search. In actuality, search is the most crucial component of cross-modal retrieval, which uses the data from one mode as the signal to access the most pertinent information from another mode. How to accurately measure the content similarity of different modal data has become a significant challenge as a result of the enormous heterogeneous gap between them [6].

RETRACTED

We live in a multimodal society, and the construction and transmission of meaning are increasingly dependent on the integration of various symbol resources [7]. Undoubtedly, in the link of English teaching, we have paid more and more attention to and used some multimodal resources, such as using nonverbal symbols, for example, visual images, sounds, colors, spaces, animations, and so on to express and communicate meanings. It can be said that a prominent part of English teaching reform is to integrate this multimodal symbol resource into our teaching methods. On the one hand, teachers use PPT courseware to teach. PPT courseware, a demonstration material compiled in the classroom, can help students to attract their attention, and improve their interest in foreign language learning, and is especially suitable for the classroom environment. On the other hand, under the guidance of the “student-centered” teaching philosophy, we emphasize students' English application ability, thus providing a stage for students to display their English application ability by using multimodal resources [8]. It can be seen that teachers are aware of the importance of using multimodal means in foreign language teaching. However, the research on multimodal teaching mode is still in the initial and exploratory stage. During the whole process, we found that there are still some problems in multimodal teaching design, which did not achieve the desired teaching effect, and made many teachers and students feel at a loss [9]. How to scientifically and effectively set up multimodal resources is helpful for teachers to successfully teach English on the multimodal stage, which has become an important topic in our English teaching reform at present. College English multimodal teaching mode is based on “students as the main body and teachers as the leading,” which makes full use of the multimodal effect, makes use of scientific and technological background and network advantages, introduces a phased evaluation system to stimulate English learning motivation, gives full play to teachers' teaching leadership, and measures the level of multimodal teaching. The construction of this teaching model reflects the sustainable teaching development direction of “teaching and learning echo, resources and environment integrate, and process and evaluation match.” Therefore, based on the multimodal discourse analysis theory, this paper first points out some existing problems by investigating and analyzing the present situation of multimodal discourse teaching in the college English classroom, and then tries to explore multimodal discourse patterns in English teaching in order to further promote college English teaching reform. This paper mainly discusses the multimodal learning algorithm based on image and text search; studies the feature extraction, relation learning, and retrieval methods of multimodal models; and transfers the more complex models to the deep learning framework. Finally, we use the public dataset to conduct image retrieval experiments, and compare it with other image retrieval work to analyze the advantages and disadvantages of the algorithm.

RETRACTED

The main contributions of this paper include the following:

1. We use the dependency-tree recurrent neural network and the bidirectional recurrent neural network to obtain text features containing sentence structure information.
2. We propose the multimodal models according to text features, and determine the use and positioning of these models according to their advantages and disadvantages.
3. A multilevel relevance learning method is proposed and applied to a cross-modal retrieval system, and uses the learned label information for semantic regularization to improve the performance of the entire cross-modal retrieval system.

## 2. Related Work

In terms of text, Guo et al. constructed a language model through a three-layer neural network due to various shortcomings of the model [10]. In this model, the features of words can be compared with each other as real-valued vectors, and the basic concepts of text are not much different from later language models. Rah and Kim introduced the constrained Boltzmann machine in the natural language model, gradually modified the energy function in the basic constrained Boltzmann machine, and finally obtained the log-bilinear model [11]. Mc et al. proposed a bimodal deep autoencoder to learn multimodal semantic relations by layer-by-layer training and joint features [12]. Penuel constructed a multimodal model by combining a convolutional neural network with a word vector model [13]. From the perspective of image-based technology generation, it is mainly based on the natural language models, introducing image features, and learning how to influence the generation probability of words according to images. Baumfalk et al. implemented text generation in a recurrent neural network-based model [14]. This paper analyzes the method of extracting features from the multimodal models based on full image and text features using the deep learning models, and proposes a multimodal feature learning method based on the characteristics of the features, but ignoring the fixed length. Functions cannot account for the complex image or sentence problems. Based on the idea of the topic model, Kelly constructed an iterative soft-maximization model by exploiting the finite properties of Boltzmann machines [15]. Liu makes full use of multimodal resources to carry out corresponding English extracurricular activities to cultivate students' multimodal reading ability [16]. Ziedonis discussed the effect of the multimodal autonomous listening teaching mode on learners' listening level and multiliteracy ability [17]. Li [18] discussed the improvement of English writing teaching from a multimodal perspective.

RETRACTED

## 3. Construction of a Multimodal Teaching Model for College English

### 3.1. Building Content

The group characteristics of college students must first be understood before building a multimodal teaching model for college English that can proceed. Students in college are different from those in high school. College students have reached the adult stage of development thanks to their extensive life experience, knowledge accumulation, and psychological maturity. They are diverse and have potentially given the evolving social environment. It also exhibits a distinct rebelliousness at the same time. English multimodal teaching is designed with college students in mind based on their characteristics. Second, we learn how to control the computer's tactile, auditory, and visual effects. College students learn English through a combination of their visual, auditory, and tactile senses. In order to accomplish the goal of college English teaching, the multimodal teaching method for college English can be used in conjunction with the physiological and psychological traits of individual college students and by fully integrating the effects of multimodal vision, hearing, and touch.

Teachers play an indispensable role in the construction of the college English multimodal teaching model. As the guide and guide of multimodal theory teaching, teachers guide students' English learning process. Therefore, college English teachers should establish multimodal teaching beliefs, adopt diversified multimodal English teaching methods, and learn more about multimodal teaching. Environmental factors can drive people's perception and behavior and improve the effect of activities in the environment.

RETRACTED

### 3.2. Main Problems in the Implementation of Multimodal Teaching

With the deepening of the multimodal teaching concept, many English teachers have begun to try to teach English knowledge and skills through various channels to improve students' multimodal communication ability and learning ability. However, multimodal teaching is more complex than single-mode teaching, which puts forward higher requirements for teachers' teaching ability and students' learning needs. Therefore, there are many problems in the process of teaching implementation. These problems are mainly reflected in many aspects. First, the teaching quality of English teachers generally needs to be improved in multimodal teaching. Many teachers' English teaching ideas and teaching methods are relatively lagging behind. They mainly carry out single-channel and single-mode teaching under the guidance of examination. Many knowledge and ability are taught to students mainly through indoctrination, which cannot realize “multimode input,” which affects students' interest in English learning. Second, students' awareness and ability of multimodal learning are relatively insufficient. Due to the long-term influence of examination-oriented education thinking, college students have an obvious tendency of “emphasizing reading and writing and neglecting listening and speaking” in English learning, whether in primary and secondary schools or in universities. They have not formed a good habit of carrying out multimodal learning. Some students even lack adaptability to the multimodal teaching mode of English. This shows that college students' awareness and ability of multimodal learning are insufficient. Finally, colleges and universities lack a good environment for the implementation of multimodal teaching. The construction standard of the English education environment in colleges and universities lags behind. English teaching is carried out in ordinary classroom most of the time, and there are few opportunities to enter high-standard voice room or multimedia classroom. On the other hand, the presentation form of English knowledge in teaching materials is relatively single, which limits the integration of various modes in the process of English teaching and is not conducive to the effective organization and implementation of college English multimodal teaching activities.

### 3.3. Multimodal Model

#### 3.3.1. Multimodal Model of Dependency-Tree Recurrent Neural Network

In a modality, when using the input features to retrieve the features in the existing data, it is hoped that the correct results will be in the earlier position in the output queue. When retrieving data, the input features can be compared with the features in the database to obtain the similarity. According to this idea, for mutual retrieval between two modes, it is also necessary that the correct results are in the forefront, and the data of different modes can be compared in similarity, so a permutation loss function is defined to complete feature fusion [19]. First of all, image features and text features are in different feature spaces, so this paper transforms image features to make their dimensions the same as text features, as shown in formula (1).

(1) $$\begin{array}{c} v_{i}=W_{I}x_{i}. \end{array}$$

*v*_*i*_ is the linearly transformed feature. If each picture corresponds to a sentence, the feature obtained through the recurrent neural network is *y*, and the permutation loss function is obtained as follows:

(2) $$\begin{array}{c} J\left(W_{I},\theta \right)=\sum_{i}\sum_{j\neq i}\max\left(0,\Delta -v_{i}^{T}y_{i}+v_{i}^{T}y_{j}\right)\\ +\sum_{j}\sum_{i\neq j}\max\left(0,\Delta -v_{j}^{T}y_{j}+v_{j}^{T}y_{j}\right). \end{array}$$

*θ* is a parameter of the recurrent neural network, and the similarity between different modal features is expressed by inner product. The first term of the loss function is to retrieve sentences according to pictures. *v*_*i*_^*T*^*y*_*i*_ in max function indicates the similarity of correct pictures and text combinations, and *v*_*i*_^*T*^*y*_*j*_ indicates the similarity between a given picture *i* and the wrong sentence *j*. According to the idea that the correct result should be in the forefront, the loss function requires that the inner product of the correct result is larger than that of the wrong result. If this condition is satisfied, then the result of max function is 0. Δ is the difference degree of inner product. The larger the Δ is, the higher the discrimination performance of the model between right and wrong is, but too large Δ will make the model unable to converge. The second term of the loss function is to retrieve the picture with a given sentence. The loss function is non-negative. If the loss function is 0, then all the correct inner products are greater than the wrong inner products. The training of the model is to minimize the loss function.

RETRACTED

A full image or sentence is used to extract a fixed-length feature, but the feature is insufficient to describe complex content [20]. As a result, the acquired features are typically directed at a specific object, making it impossible to gather information about the background and other objects or making it less obvious in the features. This issue needs to be resolved by the image part by directly extracting features from the image's objects in order to obtain more fine-grained features [21]. The text portion is similarly true, but each word vector in the text is a more fine-grained feature, with the exception that the feature does not contain information about sentence structure. This study employs hidden state transfer and a bidirectional recurrent neural network to address the issue of sentence structure. The correct object-word combination is used in this study to appear more frequently in the training data than the incorrect combination in order to address the issue of many-to-many fine-grained features, and the following similarity evaluation function is defined as follows:

(3) $$\begin{array}{c} v=W_{m}\left[{\text{CNN}}_{\theta_{c}}\left(I_{b}\right)\right]+b_{m}, \end{array}$$

(4) $$\begin{array}{c} S_{kl}=\sum_{t\in gl}\max_{i\in gk}v_{i}^{T}s_{t}, \end{array}$$

(5) $$\begin{array}{c} S_{lk}=\sum_{i\in gk}\max_{t\in gt}v_{i}^{T}s_{t}. \end{array}$$

In formula (3), after the feature is obtained from the object image *I*_*b*_ through the CNN network, the linear transformation is used to make it in the same dimension as the text feature. In formula (4), *g*_*k*_ represents the bounding box index set of the *k*-th picture, and *i* represents the *i*-th bounding box, so *v*_*i*_ represents the feature of the *i*-th bounding box in the picture; if the *k*-th picture has 20 boundaries box, then *g*_*k*_ = {1,…, 20}. Similarly, *g*_*i*_ represents the word index set of the *l* th sentence, and the similarity evaluation between features still uses the inner product. The max function is to find the bounding box corresponding to the image feature with the largest *s*_*t*_ inner product when the word *t* in the sentence is given, and to form the correspondence between the word and the object. The *S*_*kl*_ obtained by summing all the words is the similarity of the sentence *l* and the picture *k* after the sentence *l* is given and the corresponding bounding box is found for each word. Equation (4) is also used to retrieve the picture for the given sentence. Similarly, in formula (5) is given the picture *k*, and after each bounding box finds the corresponding word, the similarity between the picture *k* and the sentence *l* is obtained, which can be used to retrieve the text for the given picture. Since there is a correspondence between objects and words, such as a picture of a dog and the word “dog,” the frequency of this combination will be higher than other wrong combinations, so the model will be more inclined to associate the picture of a dog. The calculation result shows that the value of the inner product is higher.

RETRACTED

According to equations (2), (4), and (5), the permutation loss function of the fine-grained multimodal model can be obtained as follows:

(6) $$\begin{array}{c} J\left(\theta \right)=\sum_{k}\sum_{l}\max\left(0.\Delta -S_{kk}+S_{kl}\right)\\ +\sum_{k}\sum_{l}\max\left(0,\Delta -S_{kk}+S_{lk}\right). \end{array}$$

At that time, *k*=*l* represents the correct picture-text combination, and the training method of this function is the same as that of algorithm formula (1).

The multimodal data classification network framework is used to verify the effectiveness and rationality of the designed multimodal data tag cleaning and prediction network. The basic network framework is shown in Figure 1. The classification framework is similar to the overall framework of the tag cleaning framework. The data go through the same image embedding subnetwork, text embedding subnetwork, and feature fusion layer, and then the two modal data features are fused and sent to the full-connection layer. Finally, the output dimension of the full-connection layer is consistent with the data dimension of the label, and its supervision information comes from two parts: the accurate label of the artificially verified accurate label set and the predicted label obtained by the network processing of the noise label dataset.

In the multimodal data classification network framework, the feature extraction network for image data and the feature extraction network for text data have the same architecture as in the multimodal data label generation network.

*X* is output as *h*_*x*_ after using the image feature extraction network as follows:

(7) $$\begin{array}{c} h_{x}=f_{x}\left(X;W_{x}\right). \end{array}$$

Text data *Y* is output as *h*_*y*_ after passing through the text feature extraction network as follows:

(8) $$\begin{array}{c} h_{y}=f_{y}\left(Y;W_{y}\right). \end{array}$$

In the fusion layer, image data features *h*_*x*_ and text data features *h*_*y*_ are fused. The fusion process can be regarded as the process of using the Cartesian product as follows:

(9) $$\begin{array}{c} \left\{\left(h_{x},h_{y}\right)|h_{x}\in \left[\begin{array}{c} h_{x}\\ 1 \end{array}\right],h_{y}\in \left[\begin{array}{c} h_{y}\\ 1 \end{array}\right]\right\}. \end{array}$$

This definition is mathematically equivalent to image data representing *h*_*x*_ and text data representing the outer product of *h*_*y*_.

(10) $$\begin{array}{c} h_{m}=\left[\begin{array}{c} h_{x}\\ 1 \end{array}\right]⊗\left[\begin{array}{c} h_{y}\\ 1 \end{array}\right]=\left[\begin{array}{cccc} h_{x} & h_{x} & ⊗ & h_{y}\\ 1 & \; & \; & h_{y} \end{array}\right], \end{array}$$

where ⊗ represents the outer product between two vectors, and *h*_*m*_ represents all three possible combinations of two single-mode features. *h*_*x*_, *h*_*y*_ is a single-mode interaction composed of single-mode features, and *h*_*x*_ ⊗ *h*_*y*_ is a dual-mode feature interaction. This fusion can also be extended to the interaction between multiple modal data.

RETRACTED

#### 3.3.2. Multimodal Data Fusion Strategy

We cascade the features from various modal data to create the most straightforward and popular fusion method. This approach can be seen as a straightforward special case of the fusion reasoning definition given above. People frequently combine data from various modalities in order to fully utilize the complementary information provided by multimodal data, which has also emerged as a multimodal data research hotspot. The previous learning algorithm offers more flexibility in early fusion, late fusion, and mid-term fusion, which are the three categories of multimodal data fusion. Late fusion is also known as decision-level fusion, while early fusion is also known as feature-level fusion. Fusion, also known as mid-term fusion, is a continuation of feature-level fusion. Different fusion processing techniques can be chosen for various learning tasks.

Early fusion has a lot of early research in the field of multimodal data fusion, as shown in Figure 2. One of its core ideas is to integrate multiple data sources into a single feature vector and then use the fused feature vector as the input of the machine learning algorithm to adapt to a task. Early fusion is very challenging because it does not extract features from different data sources but directly integrates the original data.

Late fusion is different from early fusion in that it does not fuse the original data dimension, but trains and learns the data of each modality with different algorithm models, and fuses the different results in a certain decision-making way to get the final decision-making result, as shown in Figure 3. The advantage of late fusion is that the errors of different classifiers are often uncorrelated from each other, and the results are more accurate by choosing different models for different data.

In the later fusion strategy, it is very important to choose different neural network architecture according to the characteristics of different modal data. At this stage, the convolutional neural network is generally used for image data; the cyclic neural network is generally used for text audio and other serialized data; or in simpler cases, several fully connected layers will be selected to complete feature extraction. Then, different feature representations are fused by sharing the representation layer. The shared presentation layer here is not limited to one network layer, but refers to the common space, where the implicit correlation of various modal data can be mined. Because of the powerful modeling and feature extraction capabilities of various neural network structures and the flexibility of choosing to share the depth of the representation layer, the later fusion has better experimental results than other fusion methods and strategies.

RETRACTED

In particular, first, the current situation of noise labels in the multimodal dataset is analyzed, and aiming at the shortcomings of the existing algorithms, a noise label cleaning and prediction network for multimodal data is proposed. Then, a multimodal data classification network is designed to detect the accuracy and effectiveness of the designed label cleaning and predict the labels generated by the network. Experimental results show that the proposed method can effectively deal with the noise labeling problem in multimodal datasets.

## 4. Result Analysis and Discussion

In order to understand the current state of multimodal discourse teaching in college English classes, learners' cognition, and demands for multimodal resource setting and teaching reform in English teaching courses, we have learned about the use of multimodal resources in some English teaching classes in some colleges and universities through questionnaires and interviews. We create a questionnaire on students' opinions on the use of multimodal resources in the classroom, student behavior when using multimodal resources, and student feedback on the effectiveness of multimodal instruction that makes up the bulk of the questionnaire design. The majority of the questionnaire's questions, such as “students' attitude toward PPT courseware used in English classroom” and “students' cognitive effect of multimodal courseware PPT on English learning,” are designed with PPT as the main theme because visual and auditory modalities primarily depend on the setting and presentation of PPT courseware. In addition to PPT courseware, the open-ended questions in the questionnaire also refer to teachers' body language and other modal resources. Students in science and liberal arts, undergraduates, and graduate students participated in this survey. Comprehensive colleges, business colleges, and science and engineering colleges are all covered by the questionnaire.

Statistical Results and Analysis. First of all, the statistics of the questionnaire data show that teachers use multimodal resources in classroom teaching more frequently, and the multimodal resources used are rich and balanced, involving text, pictures, videos, etc., as shown in Figure 4.

In English classroom teaching, while teachers use PPT courseware for teaching, they will also use other multimodal resources to enrich and balance teaching, such as various body languages (as shown in Figure 5).

RETRACTED

From the results of the questionnaire, we can see that the construction of multimodal discourse plays an important role in college English class. In this multimodal discourse context, the teacher's constructive role is particularly important, and the classroom teaching discourse led and organized by the teacher is a dynamic discourse. Teachers need to strengthen the awareness of multimodal discourse construction in the classroom, and properly allocate and adjust the different modal configurations they use in the classroom according to the context; classroom multimodal discourse construction also includes instructing students to use multimodal resources in communication scenes to improve students' multimodal reading ability, especially multimodal English reading ability related to professional disciplines. Each related professional topic has its own unique structural characteristics. At present, most discourse teaching, such as the genre teaching method, mainly focuses on the interpretation of text discourse, ignoring the meaning construction of other modes. In fact, all potential meanings are multimodal, and discourses of different disciplines will involve images and images.

We follow a two-stage optimization strategy when learning the entire cross-modal retrieval system model. Because if the image embedding network and the text embedding network are learned at the same time, the whole optimization process may become oscillating or divergent. Therefore, it is recommended that different modal data networks are separately trained and then unified for fine-tuning. We follow a similar strategy when training the model, first learning the model weights for the image network, then learning the model weights for the text network, and finally, fine-tuning the two together.

Our experiments are mainly used to test two directions: one is the specific improvement effect of the proposed multilayer correlation mining method on cross-modal retrieval experiments; the second is to verify the specific semantic information contained in tags in cross-modal retrieval experiments' effect.

Evaluation criteria are as follows: *R*@*K* and MAP, (1,10,20) are used as the experimental simulation criteria in this section.

*R*@*K*: it refers to the proportion of correct results among the first *k* results retrieved. For example, we have 100 test samples, and 80 samples in the actual retrieval results can find the correct matching results from the top 10 results retrieved by the algorithm, so the *R*@10 is 80/100∗100% = 80%, so in the actual evaluation criteria, the larger the value, the better the actual algorithm retrieval results. Map: MAP (mean average precision) is a commonly used cross-modal retrieval index.

RETRACTED

Flickr8k dataset: Flickr8k dataset contains 8000 pictures collected from different Flickr groups. Each picture corresponds to five sentences describing the content of the picture. These sentences are independently written by native English speakers. Flickr8k dataset does not classify the image text content in any way.

Flickr30k dataset: Flickr30k dataset is an extension of the Flickr8k dataset. This dataset contains a total of 31783 images, which generally focus on events involving people and animals. Each picture corresponds to five statements describing the content of the picture. Similarly, the Flickr30k dataset does not classify the text content of the picture.

Table 1 shows the results of the multilayer correlation mining method and the other cross-modal retrieval methods on the Flickr8k dataset.

Table 2 is a comparison between the results of the multilayer correlation mining method and the other cross-modal retrieval methods on the Flickr30K dataset.

Figure 6 shows the performance of the proposed cross-modal retrieval algorithm on the Flickr8k dataset test set with the increase in the number of iterations:

Figure 7 shows the performance of the proposed cross-modal retrieval algorithm on the Flickr30K dataset test set as the number of iterations increases.

From the above experimental results, we can see that compared with the MCNN method, on the Flickr8K dataset, the R@10 retrieval index of our proposed method is improved by about 0.8% in the image retrieval experiment and about 1.6% in the sentence retrieval experiment. On the Flickr30K dataset, the retrieval index of R@10 is improved by about 1.2% in the image retrieval experiment and about 2.6% in the sentence retrieval experiment. Therefore, whether in the experiment of image retrieval text or text retrieval image, our method has achieved good experimental results. This further confirms our view that the relevance of multimodal data is not limited to the semantic features of a certain layer, and fully exploiting the multilevel relevance will positively improve the actual effect of cross-modal retrieval. This multilevel concept can also be extended to other multimodal data learning algorithms. For example, realizing layer-by-layer fusion in multimodal data fusion will also be helpful to specific learning tasks.

This experiment is used to test the effectiveness of the proposed method. By testing the actual effect of classification on the test set, the quality of the labels generated by the proposed method is judged. In addition, the classification performance of unimodal data and multimodal data is also tested. The performance of the proposed algorithm on the test set is shown in Figure 8.

RETRACTED

From the above experimental results, we can see that: compared with the single-mode data experiment, the multimode data use more complementary information of modal data, so the classification accuracy is higher; at the same time, the effect of learning directly using the noise label multimodal dataset is relatively poor. The noise label will interfere with or mislead the classification network to recognize and distinguish the data.

This section mainly studies the performance of the cross-modal retrieval method of image text on the Flickr8K dataset and Flickr30K dataset. It focuses on how to more effectively mine the correlation between different modal data and establish a multimodal data retrieval method. Multiple feature output channels are then used for correlation mining at different feature layers. Finally, various objective loss functions are used and combined to drive the learning and convergence of the entire model parameters. The experimental results show that multilevel correlation mining is beneficial to improve the performance of the cross-modal retrieval system. In addition, through the semantic regularization of label information, the correlation mining in the modal data is completed, which further improves the performance of the cross-modal retrieval system.

## 5. Conclusions

The multimodal discourse analysis theory is the foundation of this study. We are able to comprehend the use of multimodal resources in English teaching through a more thorough, in-depth, and methodical investigation. In addition to conducting preliminary research on dynamic multimodal discourse in college English classroom teaching, this paper discusses the construction content of multimodal teaching mode, deepening the understanding of multimodal discourse analysis in educational reform through discourse research. The effective use of multimodal noise label data for multimodal learning is suggested. In order to learn the mapping knowledge from the noise feature space to the accurate semantic label space, this method makes use of a small subset of human-verified accurate labels in the multimodal dataset, removing the remaining noisy labels and making predictions. The multimodal data classifier is used to test the effectiveness of the proposed network, and the multimodal data noise label cleaning and prediction network is the main component of the method's overall framework. The multimodal data fusion layer, image embedding subnetwork, text embedding subnetwork, numerous fully connected layers and nonlinear transformation layers are the main modules in the network. The primary benefit of this approach is that the network structure is simple, the noise label data can be processed more efficiently, and better task results can be obtained than with a machine learning algorithm applied directly to the original noise label data. The multimodal model has its limitations, too. The depth of different modal data research places restrictions on multimodal models. For instance, the multimodal model can further learn these features and produce better results. The application of deep learning in pictures, text, and speech has made great progress in these types of feature extraction. Additionally, the multimodal model currently does not use more modal data. The learning parameters will also increase as the modes do. In addition, it is necessary to investigate whether adding more modal data can enhance performance. The model will not be able to converge if there are too many modes.

RETRACTED

The multimodal data learning algorithm based on image and text retrieval has produced some theoretical and experimental results in this paper, but there are some limitations because of the time and skill constraints on some of the research. In this paper, a method for performing other machine learning tasks is proposed that involves first processing noise labels. Future research may focus on algorithms that are specifically resistant to noise labels. For noise labels, the two might work better together. With more sophisticated feature extraction techniques for various modal data, particularly text data, the cross-modal retrieval algorithms are becoming increasingly accurate. In the future, you can experiment with various processing techniques or employ graph neural networks. The text modal data's internal connections are further explored by the network.

## Figures and Tables

**Figure 1:** Multimodal data classification network.

**Figure 2:** Early fusion.

**Figure 3:** Late fusion.

**Figure 4:** Multimodal resources in English classroom teaching courseware.

**Figure 5:** Other multimodal resources in English classroom teaching.

**Figure 6:** Performance chart of the proposed algorithm on Flickr8K dataset test set.

**Figure 7:** Performance of the proposed algorithm on the Flickr30k dataset test set.

**Figure 8:** Performance of the proposed algorithm on the test set.

**Table 1:** Comparison of performance of cross-modal retrieval methods in Flickr8K dataset.

Algorithm model	Image retrieval			Sentence retrieval		

R@K	1	10	20	1	10	20
Random ranking	7.1	15.6	19.8	6.9	14.9	20.3
SDT-RNN	5.9	20.1	23.2	4.8	31.7	27.3
Deep fragment	6.6	29.6	30.9	6.0	22.7	34.1
MCNN	20.3	21.6	42.5	24.7	12.6	54.2
Proposed	25.6	35.7	56.8	28.3	44.7	62.2

RETRACTED

**Table 2:** Performance comparison of the cross-modal retrieval methods on Flickr30K dataset.

Algorithm model	Image retrieval			Sentence retrieval		

R@K	1	10	20	1	10	20
Random ranking	7.1	15.6	19.8	6.9	14.9	20.3
SDT-RNN	7.5	25.3	26.7	6.9	34.7	40.2
Deep fragment	8.1	36.9	49.3	10.1	35.7	46.3
MCNN	26.3	29.6	49.1	29.3	18.5	67.1
Proposed	32.1	49.2	72.3	37.9	65.1	75.5

## Data Availability

The data used to support the findings of this study are available from the corresponding author upon request.
